This article has been retracted.

# Effect of Mosaic Allograft Osteochondral Transplantation Combined with Corrective Osteotomy in Treating Osteochondral Lesions of the Talus on Ankle and Knee Joint Function and Lower Limb Alignment

**DOI:** 10.1155/2022/9688098

**Published:** 2022-07-15

**Authors:** Zhenshuan Zhao, Jun Li, Xiaoguang Yu, Guobin Liu, Feng Zhao, Ruiqi Li

**Affiliations:** Department of Orthopaedics, The First Hospital of Hebei Medical University, Shijiazhuang, Hebei 050000, China

## Abstract

**Objective:**

To explore the effect of mosaic allograft osteochondral transplantation combined with corrective osteotomy in treating osteochondral lesions of the talus (OLT) on ankle and knee joint function and lower limb alignment.

**Methods:**

One hundred and thirty-three OLT patients treated in our hospital between July 2015 and October 2019 were enrolled. Regarding the various surgical approaches, they were categorized into two groups, namely, A and B including 69 and 64 cases, respectively. The patients in group A were processed with mosaic allograft osteochondral transplantation combined with corrective osteotomy, and the patients in group B were processed with microfracture surgery. The Baird ankle function score and visual analog scale (VAS) were employed for evaluating the surgical efficacy and the degree of pain prior to and following surgery. The pre- and postoperative surgery-related indicators, Ankle Hindfoot Scale (AOOFAS), HSS score, lower limb alignment, and range of motion of the ankle were compared between the two groups, and changes in growth factor levels prior to and following processing were observed.

**Results:**

Overall scores were better in group A than in group B (*P* < 0.05). The operation length was longer in group A, the amount of intraoperative blood loss was greater, and the length of hospitalization was less than in group B. The VAS score 48 hours after surgery was also lower (*P* < 0.05). Postoperative AOFAS scores in group A were better, and lower limb alignment was also less than in group B (*P* < 0.05). The postoperative HSS score did not differ significantly between the two groups (*P* > 0.05). The range of plantar flexion and dorsiflexion of the ankle joint was better in group A, and the levels of endothelial growth factor (VEGF), platelet-derived growth factor (PDG), and transforming growth factor *β*1 (TGF-*β*1) were lower than those in group B (*P* < 0.05). The occurrence of postoperative problems did not differ between the groups (*P* > 0.05).

**Conclusion:**

Mosaic allograft osteochondral transplantation combined with corrective osteotomy has a high effective rate in the treatment of OLT, which can promote the healing of articular cartilage and the recovery of ankle joint functions, improve the range of motions of the ankle, and improve the lower limb alignment.

## 1. Introduction

Osteochondral lesions of the talus (OLT), also known as osteochondritis dissecans of the talus, is a common cartilage damage disease, which occurs in both acute and chronic ankle injuries. The main manifestations of the patients are local articular cartilage exfoliation and mostly involving the deep subchondral bone [1, 2]. Relevant studies have pointed out that the nutrition of cartilage mainly depends on flow of joint synovial fluid, which may affect its self-repair ability after injury and eventually lead to the formation of bone cyst [3]. The primary goal of OLT therapy is to create stable cartilage relief, eliminate pain, and restore ankle function. At present, conservative treatment, surgical treatment, or both are used for treatment. OLT treatment includes arthroscopic debridement, microfracture and drilling, reduction and internal fixation, autologous or allogeneic osteochondral graft, and autologous periosteum graft. Microfracture treatment for OLT is the first surgical treatment after the failure of conservative treatment. Compared with invasive surgery, bone marrow stimulation is widely used because of its low trauma, low complications, good postoperative effect, simple operation, and low cost. The operation time of ankle microfracture under arthroscopy is short, which can rapidly improve the speed of tissue repair of patients. It is suitable for cartilage injury with slight damage of articular surface. The procedure is simple, requiring less than 1 h of operation and 1 d of hospital stay. Compared with traditional surgery, it can preserve the integrity of the subchondral plate and avoid changing the physical properties of the articular surface and damaging the mechanical support structure. However, according to relevant reports, some patients still do not get ideal therapeutic effect after receiving microfracture treatment [4]. Osteochondral grafting, including autograft and allograft, is a better option for treating large OLT patients with full-thickness articular cartilage damage, with or without subchondral bone cysts. The donor sites for autotransplantation are usually osteochondral from non-weight-bearing areas such as the medial side of the knee or the lateral malleolus of the femur. The objective of osteochondral transplantation is to reconstruct the mechanical, structural, and biochemical properties of hyaline cartilage in the injured joint. Selection of osteochondral graft donors. Studies have pointed out that autologous bone transplantation is able to successfully ameliorate the surgical effectiveness of patients with OLT [5]. Due to the limited source of autologous cartilage in patients and its influence on the structure and function of donor site, allogeneic osteochondral graft materials are relatively easy to obtain, with unlimited size and shape, and have biological activity. They can undergo biological healing with the recipient part, while retaining attachment points of muscles, ligaments, and joint capsules [6]. Therefore, in this study, mosaic allograft osteochondral transplantation was used for treatment. The lower limb alignment is defined by the line drawn between the mechanical axes of the tibia and femur. Clinical data show that poor lower limb alignment can accelerate the development of varus and valgus deformity of knee joints [7]. It has also been reported that poor lower limb alignment can aggravate the wear degree of ankle joint and medial knee joint and affect postoperative recovery [8]. However, the research on the effect of mosaic allograft osteochondral graft combined with corrective osteotomy on the recovery of lower limb alignment in OLT patients is still in the exploratory stage. Therefore, the current exploration is aimed at exploring the influences of combined treatment of OLT on ankle and knee function and lower limb alignment and providing reference for the selection of treatment options for this disease.

## 2. Materials and Methods

### 2.1. Clinical Data

This study was a retrospective study. One hundred and thirty-three OLT patients, including 77 men and 56 women, treated in our hospital between July 2015 and October 2019 were enrolled. The average age was 52.47 ± 7.38 years; the mean bone loss area under MRI was 2.12 ± 0.5 cm^2^; and the mean course of disease was 3.65 ± 0.61 months. Among them, 12 patients were complicated with diabetes, 23 sufferers with hypertension, and 14 sufferers with coronary heart disease. Sixteen sufferers had a background of fracture. This survey was confirmed through the ethics committee of our hospital on January 5, 2020.

### 2.2. Inclusion Criteria

The inclusion criteria were as follows: (1) patients fulfilled the OLT diagnostic criteria [9]; (2) patients signed the informed consent form; (3) unilateral OLT; (4) patients underwent surgical treatment; and (5) patients with complete clinical data.

### 2.3. Exclusion Criteria

The exclusion criteria were as follows: (1) patients with severe coagulation abnormality; (2) patients with other ankle joint diseases; (3) cartilage injury was more than 10 mm; (4) patients with fractures in other parts; (5) patients with severe osteoarthritis; (6) patients with severe bone and joint ligament injury; (7) patients with bleeding disorders; and (8) patients with traumatic arthritis.

### 2.4. Methods

1. Group A was treated with mosaic allograft osteochondral transplantation combined with corrective osteotomy. (1) Allograft bone extraction: before implantation, the individualized shaping of the grafted bone block was carried out according to the three-dimensional space of the talus defect. The bone block was drilled with Kirschner wire or fine drill for mesh treatment. PRP solution was applied to infiltrate the allograft bone block to promote bone healing. (2) Mosaic allograft osteochondral transplantation combined with corrective osteotomy: the patient was located in a supine situation, a balloon tourniquet was applied, and the pressure was set to 45 kPa. The medial or posteromedial surgical approach of the affected ankle joint was chosen in accordance with the injury site. The length of incision was about 5 cm, and the medial malleolus and ankle mortise were exposed. Two Kirschner nails were driven into the medial malleolus as ankle nail fixation markers. Kirschner nails were removed, osteotomy was performed with a pendulum saw, and talus was exposed. Oblique osteotomy was performed at 2.5 cm near the tip of the medial malleolus for the medial injuries, and lateral malleolus fibula osteotomy was performed for the lateral injuries. Under arthroscopy, the diseased cartilage and subchondral bone were excised to normal bone tissue, keeping the flat base of the lesion. The operation was carried out according to the guided drilling, which was at right angles to the surrounding soft tissue wall, and the appropriate guide drilling was selected according to the lesions. The grafted bone was lightly beaten with a stick to make the cartilage surface of the grafted bone parallel to the cartilage surface of talus, and the large gap between the grafted bone blocks was filled with cancellous bone slices. (3) Postoperative treatment: plaster immobilization was performed for 3 weeks following the operation, and non-weight-bearing exercise activities began. Partial weight-bearing activities could be carried out 5 weeks later, and weight-bearing activities could be carried out 8 to 12 weeks later
2. Group B was treated with microfracture surgery, and MRI was used to measure the maximum length and width of the damaged area before surgery to calculate the cartilage damaged area. Lumbar spinal anesthesia was performed, the patient was located in a supine situation, and a tourniquet was applied to the affected thigh to stop the bleeding. Ankle arthroscopy was used to observe the hyperplasia of the ankle joint and joint synovium. Anteromedial and anterolateral approaches were selected in accordance with the patient's circumstance. The anterolateral approach is located at the intersection of the external end of the ankle joint line with the third peroneal muscle, and the anterolateral approach is located at the intersection of the medial side of the tibialis anterior tendon with the articular line and the lateral side of the saphenous vein and nerves. The hyperplasia synovium and necrotic cartilage and granulation tissue were removed with a curette and scalpel, and vertical holes were perforated on the cartilage defect site and subchondral bone plate of talus with microfracture instruments, and then, the tourniquet was relaxed. The postoperative treatment was the same as group A

### 2.5. Observation Indicators

The observation indicators as follows: (1) clinical efficacy: Baird-Jackson ankle function score was used to evaluate the surgical efficacy [10]. The score mainly included 3 dimensions and 7 items, and the score ranged from 0 to 100 points, 96 to 100 points were classified as excellent, 91–95 points as good, 80–90 points as general, and 0–80 points as poor. The rate of excellent and good scores was calculated as the (number of excellent cases + number of good cases)/total cases∗100%. (2) Operation-related indicators: length of hospitalization, operative time, and intraoperative blood loss. (3) Pain degree: pain before surgery and 24 h, 48 h, and 7 days after surgery was scored using the visual analog scale (VAS) [11]. A ruler with a length of 10 cm was used to judge, with 0 point demonstrating no pain and 10 points demonstrating severe pain. (4) Ankle and knee joint: for comparison, knee and ankle functions were assessed before and after surgery. HSS knee joint function score and Ankle Hindfoot Scale (AOOFAS) were used to evaluate the knee and ankle joint functions [12, 13]. HSS scores ranged from 0 to 100 points, with higher scores indicating better knee joint function. AOFAS scores (range 0–100 points) mainly include pain (40 points) and function (10 points) with higher scores indicative of better ankle function. A score > 75 points indicates good ankle function. (5) Lower limb alignment: the lower limb alignment is the hip-knee-ankle angle (HKA), namely, the difference between 180° and the medial angle between the mechanical shafts of the femur and tibia. Medical X-ray photography system was used for detection, and X-ray films were taken before and after surgery. The patient was photographed in a standing position with weight bearing, hands drooping, feet parallel with shoulder width, and patella facing straight forward. (6) Range of motions of the ankle joint: the range of motion of the ankle joint was measured 1 day before surgery and 3 months after surgery by Konica CR-150 X-ray machine and special data workstation. Both orthographic and lateral X-rays were used to determine the neutral position of the ankle joint. The range of plantar flexion and dorsiflexion of the ankle joint was measured based on the neutral position of the tibial axis of the ankle joint. (7) Growth factor levels: blood (3 ml) was collected after fasting on the day before surgery and three months after surgery. The serum was separated by centrifugation. An automatic biochemical analyzer was used, and the levels of endothelial growth factor (VEGF), transforming growth factor *β*1 (TGF-*β*1), and platelet-derived growth factor (PDG) were determined through double-antibody sandwich enzyme-linked immunosorbent assessment. Kits were provided by Sangon Bioengineering Co., Ltd. (8) Complications: the incidence of complications including wound infection, local swelling, poor wound healing, and osteophyte hyperplasia in the two groups was counted 3 months after surgery

### 2.6. Statistical Processing

SPSS 22.0 was used for data analysis. Categorical data were expressed as percentages, and the *χ*^2^ test was used to determine between-group differences. Results were presented as *x* ± *s* after assessment of normality distributions and homogeneity of variance and analyzed by *t*-tests. *P* < 0.05 indicated statistical significance.

## 3. Results

### 3.1. Comparison of Patient Characteristics between the Two Groups

The groups did not differ significantly (*P* > 0.05), as shown in Table 1.

### 3.2. Effectiveness of Surgery

The rate of “excellent” and “good” scores for surgical outcomes was significantly better in group A compared with group B (*P* < 0.05) (Table 2).

### 3.3. Operation-Related Indicators of the Two Groups

The duration of surgery was longer in group A, with greater intraoperative blood loss and shorter duration of hospitalization (*P* < 0.05) (Figure 1).

### 3.4. Comparison of VAS Scores before and after Surgery

There was no significant difference in the VAS scores in the two groups before surgery, after 24 h, and after seven days (*P* > 0.05). However, the mean VAS score of group A 48 h after surgery was lower than that of group B (*P* < 0.05) (Figure 2).

### 3.5. Comparisons of Ankle and Knee Joint Function and Lower Limb Alignment

No significant differences between the groups were observed in terms of preoperative HSS and AOFAS scores and lower limb alignment (*P* > 0.05). Both HSS and AOFAS scores showed improvement after surgery, with greater improvement seen in the AOFAS scores in group A (*P* < 0.05). The postoperative lower limb alignment was lower than that before surgery in both groups, while the change was more marked in group A (*P* < 0.05) (Figure 3).

### 3.6. Comparison of Range of Motion of Ankle before and after Surgery

No significant differences in the range of plantar flexion and dorsiflexion of the ankle were observed between the two groups (*P* > 0.05). The postoperative range of motion of ankle in both groups was higher than the preoperative value, with a greater change seen in group A (*P* < 0.05) (Figure 4).

### 3.7. Comparison of Growth Factor Levels between the Groups before and after Surgery

The preoperative PDG, VEGF, and TGF-*β*1 levels did not differ significantly between the two groups (*P* > 0.05). The postoperative PDG and VEGF levels in both groups were higher than those before surgery, with the levels in group A being higher than those in group B (*P* < 0.05). TGF-*β*1 levels were lower after surgery, with values in group A lower than those in group B in the two groups and lower than those before surgery, and those in group A were lower than those in group B (*P* < 0.05) (Figure 5).

### 3.8. Comparison of Postoperative Complications

The groups did not differ significantly in the incidence of postoperative complications (*P* > 0.05) (Table 3).

## 4. Discussion

OLT is the defect of articular cartilage and subchondral bone of talus vault, which is mainly related to the occurrence of traumatic events [14]. For patients who failed conservative treatment, arthroscopic debridement, scratching, microfracture, and allograft osteochondral transplantation are commonly used in the treatment of OLT. Currently, microfracture is mostly used for treatment. Through drilling through subchondral bone and draining blood, mesenchymal stem cells in the bone marrow migrate to the cartilage defect, which has a good short-term effect, but its application scope is limited, and some patients are prone to poor prognosis [15, 16]. The main problem of autologous osteochondral transplantation is the limited source, which may cause osteochondral injury and other related complications at the donor site. Zhou et al. [17] performed allograft osteochondral transplantation for OLT patients and found that this method could improve the therapeutic effect to a certain extent. In allogeneic bone therapy, allogeneic bone of an appropriate size is transplanted to the injured site, which can improve cartilage injury. In addition, bone marrow interstitial stem cells in allogeneic bone can differentiate into osteoblasts under certain induction factors, promoting osteogenesis without affecting bone tissue development [18]. The advantage of allogeneic osteochondral transplantation is that sufficient grafts can be obtained for the damaged area of the talus, and there is the possibility of a second autologous or allogeneic osteochondral transplantation if the initial operation fails. However, possible immune rejection, lower cartilage viability, longer healing period, and higher cost are also limitations and disadvantages of this technique. In addition, compared with autologous osteochondral graft, allograft osteochondral graft could be employed for large cartilage defects without the limitation of donor area and can avoid iatrogenic injury to patients [19]. The findings showed that the rate of “excellent” and “good” scores in group A was higher and the length of hospitalization was shorter than in group B, illustrating the high efficiency of mosaic allograft osteochondral transplantation combined with corrective osteotomy in the treatment of OLT. The reason is that arthroscopic mosaic allograft osteochondral transplantation can restore the joint surface curvature and support, and computer-assisted osteotomy guide plate for osteotomy can improve the mechanical environment and thus improve the surgical efficacy [20]. In addition, this study found that the operation time was longer in group A, accompanied by greater intraoperative blood loss, indicating that compared with microfracture, the mosaic allograft osteochondral transplantation combined with corrective osteotomy can diminish the time of operation and decrease the amount of intraoperative blood loss. However, clinical studies have found that immune rejection may occur during allograft osteochondral transplantation [21]. Therefore, in this study, the antigenic structure of allogeneic bone cells was destroyed by cryogenic treatment before allograft osteochondral transplantation, thus reducing antigenicity. Deep cryopreservation can destroy the antigenic structure of cell surface, but it can greatly reduce the antigenicity and reduce the rejection after transplantation. Dendritic cells are an important professional antigen-presenting cells, and their antigen-presenting ability is much stronger than other antigen-presenting cells such as B cells. Deep cryopreservation selectively kills dendritic cells related to rejection, thus reducing organ transplant rejection.

OLT can cause chronic ankle pain in patients, and postoperative pain can also increase local pain, which can prolong the time for patients to get out of bed after surgery and affect surgical recovery. Relevant reports indicate that the selection of appropriate surgical methods can not only improve the surgical efficacy but also relieve pain [22]. It was also found that the group A VAS scores were lower than those of group B at 48 hours after surgery, indicating that this surgical treatment can reduce postoperative pain, but the specific mechanism is still unknown, so further analysis is needed later.

Ankle joint is a joint with large bearing capacity, and cartilage of talus trochlear articular surface is vulnerable to damage. OLT is more common in foot and ankle injuries, and patients usually present with long-term chronic pain and ankle swelling, accompanied by ankle bounce, limited range of motion, etc. [23]. The main purpose of the current OLT therapy is to create stable cartilage relief, eliminate pain, and restore ankle function. Relevant studies have indicated that appropriate surgical treatment of OLT based on patients' conditions can effectively improve ankle joint function [24]. The lower limb alignment is the angle between the mechanical axes of the femur and tibia. Relevant studies have pointed out that the analysis of the lower limb alignment of the knee joint and ankle joint before and after ankle surgery is helpful to find and improve the poor lower limb alignment, which is conducive to promoting ankle joint recovery [25]. The findings of the present research showed that postoperative AOFAS scores were higher in group A, the lower limb alignment was lesser than that of group B, and the postoperative plantar flexion range of the ankle joint and dorsiflexion range of the ankle joint were both superior to those of group B, indicating that the mosaic allograft osteochondral transplantation combined with corrective osteotomy can effectively improve ankle function and range of motion in the treatment of OLT, which is the main factor that this method can improve the surgical efficacy. The reason is that during the treatment of cartilage injury by allograft bone transplantation, the cystic cavity of the lesion should be cleaned before implantation and the chondrocytes covered, which can promote the rapid growth of chondrocytes, thus promoting the repair of cartilage synovial membrane and improving the ankle joint functions of patients [26, 27]. In the current research, it was discovered that the postoperative levels of PDG and VEGF were higher in group A while the level of TGF-*β*1 in comparison with group B, illustrating that the surgical treatment could promote the growth of cartilage and bone. This is mainly related to the repeated scouring of the intramedullary tissue by the medullary cavity brush after freeze-thaw in the mosaic allograft osteochondral transplantation combined with corrective osteotomy, so as to reduce the rejection caused by immune allergens and promote the growth of articular cartilage. Besides, the incidence of postoperative complications did not differ significantly between the groups, indicating that this was not affected by the surgical method used.

In conclusion, mosaic allograft osteochondral transplantation combined with corrective osteotomy is highly effective in the treatment of OLT, which can promote the healing of articular cartilage and the recovery of ankle function, improve the range of motions of the ankle joint, and improve the lower limb alignment. This provides a theoretical basis for clinical application and can be taken into consideration by orthopedic surgeons when choosing treatment modalities. At present, the research on the effect of Mosaic allogeneic osteochondral transplantation combined with supratalar osteotomy on the recovery of lower limb force line in OLT patients is still in the exploratory stage, and there is still a lack of relevant research. There are still shortcomings in this study. The overall follow-up period is short, which makes it impossible to assess the influence of this operation on the long-term prognosis of patients. Besides, the sample size in this study was relatively small, and prospective investigations with larger sample sizes should be undertaken in the future to confirm the accuracy of the results of this study.

## Figures and Tables

**Figure 1:** Comparison of surgery-related indicators (note: ∗ indicates significant differences (*P* < 0.05) in surgery duration, intraoperative blood loss, and duration of hospitalization).

**Figure 2:** Comparison of VAS scores before and after surgery (note: ∗ indicate significant difference (*P* < 0.05) between the groups).

**Figure 3:** Comparisons of ankle and knee joint function and lower limb alignment (note: # indicates *P* < 0.05 compared with preoperative score in the same group; ∗ indicates *P* < 0.05 for comparison with group B after surgery).

**Figure 4:** Comparison of range of motion of the ankle between the groups before and after surgery (note: # indicates *P* < 0.05 in comparison with the same group before treatment; ∗ indicates *P* < 0.05 in comparison with group B after treatment).

**Figure 5:** Levels of growth factors before and after surgery (note: # indicates *P* < 0.05 in the same group before surgery; ∗ indicates *P* < 0.05 for comparisons between the groups after surgery).

**Table 1:** Comparison of patient characteristics.

Item	Group A (*n* = 69)	Group B (*n* = 64)	*χ* ^2^/*t* value	*P* value
Gender			0.469	0.494
Male (*n*)	38	39		
Female (*n*)	31	25		
Age (years)	53.52 ± 6.07	51.29 ± 7.34	1.915	0.058
Bone loss area under MRI (cm^2^)	2.09 ± 0.41	2.16 ± 0.43	0.961	0.338
Disease duration (months)	3.56 ± 0.59	3.74 ± 0.61	1.730	0.086
Complicated with diabetes (*n*)	7	5	0.220	0.639
Complicated with hypertension (*n*)	13	10	0.240	.624
Complicated with coronary heart disease (*n*)	8	6	0.174	0.677
History of fractures (*n*)	9	7	0.139	0.709

**Table 2:** Comparison of surgical outcomes (cases, %).

Group	*n*	Excellent	Good	General	Poor	Rate of “excellent” and “good” scores
Group A	69	25	31	10	3	81.16
Group B	64	18	24	15	7	65.63
*χ* ^2^						4.132
*P*						0.042

**Table 3:** Comparison of postoperative complications (cases, %).

Group	*n*	Wound infection	Local swelling	Osteophyte hyperplasia	Poor wound healing	Overall incidence
Group A	69	1	0	0	1	2.90 (2/69)
Group B	64	0	1	1	1	4.69 (3/64)
*χ* ^2^						0.294
*P*						0.588

## Data Availability

The labeled dataset used to support the findings of this study is available from the corresponding author upon request.
